The article "Contribution of Illicit Drug Use to Pharmaceutical Load in the Environment: A Focus on Sub-Saharan Africa" was published in 2022. Journal: J Environ Public Health.

# Contribution of Illicit Drug Use to Pharmaceutical Load in the Environment: A Focus on Sub-Saharan Africa

**DOI:** 10.1155/2022/9056476

**Published:** 2022-06-08

**Authors:** Asha S Ripanda, Mwemezi J. Rwiza, Elias Charles Nyanza, Revocatus L. Machunda, Said Hamadi Vuai

**Affiliations:** ^1^Department of Chemistry, College of Natural and Mathematical Sciences, University of Dodoma, P.O. Box 338, Dodoma, Tanzania; ^2^School of Materials, Energy, Water and Environmental Sciences, The Nelson Mandela African Institution of Science and Technology, P.O. Box 447, Tengeru, Arusha, Tanzania; ^3^School of Public Health, Catholic University of Health and Allied Sciences, P.O. Box 1464, Mwanza, Tanzania; ^4^Department of Community Health Sciences, University of Calgary, Calgary, Canada

## Abstract

Illicit drug abuse and addiction are universal issues requiring international cooperation and interdisciplinary and multisectoral solutions. These addictive substances are utilized for recreational purposes worldwide, including in sub-Saharan Africa. On the other hand, conventional wastewater treatment facilities such as waste stabilization ponds lack the design to remove the most recent classes of pollutants such as illicit drug abuse. As a result, effluents from these treatment schemes contaminate the entire ecosystem. Public health officials are concerned about detecting these pollutants at alarming levels in some countries, with potential undesirable effects on aquatic species and increased health hazards through exposure to contaminated waters or recycling treated or untreated effluents in agriculture. Contaminants including illicit substances enter the environment by human excreta following illegal intake, spills, or through direct dumping, such as from clandestine laboratories, when their manufacturer does not follow accepted production processes. These substances, like other pharmaceuticals, have biological activity and range from pseudopersistent to highly persistent compounds; hence, they persist in the environment while causing harm to the ecosystem. The presence of powerful pharmacological agents such as cocaine, morphine, and amphetamine in water as complex combinations can impair aquatic organisms and human health. These compounds can harm human beings and ecosystem health apart from their low environmental levels. Therefore, this article examines the presence and levels of illicit substances in ecological compartments such as wastewater, surface and ground waters in sub-Saharan Africa, and their latent impact on the ecosystem. The information on the occurrences of illicit drugs and their metabolic products in the sub-Saharan Africa environment and their contribution to pharmaceutical load is missing. In this case, it is important to research further the presence, levels, distribution, and environmental risks of exposure to human beings and the entire ecosystem.

The article "Contribution of Illicit Drug Use to Pharmaceutical Load in the Environment: A Focus on Sub-Saharan Africa" was published in 2022. Journal: J Environ Public Health.

## 1. Introduction

The problem of drug abuse is acute worldwide, and it threatens people's lives and ecosystem sustainability. According to the United Nations Office on Drugs and Crime (UNODC) (2020) projections, 269 million persons abused substances globally in 2018, exaggerated by 30% from 2009, and over 35 million people suffer from substance use disorders [1, 2]. Although the full impact of COVID-19 on the drug market is not yet determined, the pandemic's border and other limitations have already resulted in drug shortages, resulting in higher costs and lower purity, which magnify drug problems. People who are socially and economically disadvantaged are more likely to develop drug use disorders. While drug usage is more prevalent in industrialized countries than in developing countries and affluent parts of society are more affected, drug use disorders are more common in socially and economically disadvantaged individuals [1, 2]. This may be contributed by eating habits, as the effects of the drug depend on multiple factors such as genetics, health, age, dose, and stomach contents. Only one in every eight people who require drug treatment receives it.

On the other hand, only one out of every five patients in recovery clinics is a woman, despite one out of every three drug users being a woman [1, 2]. Half of the 11 million injecting drug users are infected with hepatitis C, and 1.4 million are infected with HIV. Apart from worldwide drug control measures, amphetamine seizures increased between 2009 and 2018, though global precursor control improved [2, 3]. On the other hand, traffickers and producers turn to designer compounds to synthesize amphetamine, methamphetamine, and ecstasy to avoid international restrictions [1, 2, 4]. At the same time, with stringent measures and the need to get high without legal constraints, drug abusers are shifting from controlled substances of abuse to designer drugs [1]. Traditional misused substances such as heroin and cocaine continue to be produced at some of the greatest levels ever seen in the modern history. The rise in international drug supply and petition complicates law enforcement efforts, intensifies health hazards, and makes it more difficult to prevent and treat substance use disorders [2]. The need for drug traffickers to get a higher profit causes the observed trend of increased accessibility to novel psychoactive substances (NPS). Technical synthesis of these substances is easier, at a low cost and easier conversion to varieties by substitution, which are undetectable by current standard toxicological screens [2], which help to avoid the law prohibiting their sales and use [5–8].

The article "Contribution of Illicit Drug Use to Pharmaceutical Load in the Environment: A Focus on Sub-Saharan Africa" was published in 2022. Journal: J Environ Public Health.

Illicit drugs reach the environment mainly through human excreta. Unmetabolized parent substances and their metabolites are released in high quantities into residential wastewater via urine or faeces [5, 9]. Based on conducted studies, reports of occurrences of methamphetamine, amphetamine, morphine, MDMA, and metabolites of cocaine such as benzoylecgonine and ecgonine methyl ester are reported to be the most prevalent deposits in effluents [5, 10], indicating the possibility of a regular occurrence in surface waters than other chemicals [5]. Drugs such as morphine, amphetamines, and MDMA have significant biological actions, and their presence as complex combinations in the environment may be hazardous and poses dangers to human health and the aquatic ecosystem, despite relatively low environmental concentrations [9, 11–13]. Apart from the reported effects of these illicit substances, residues, and their transformation products on the environment [9, 11–13], there are no recommended limits for permissible quantities of these compounds in surface water, tap/drinking water, or wastewater. However, more work is needed to give a clearer picture and accurate risk assessment.

Apart from all of these facts, there are 17 agreed-upon sustainable development goals to be met by 2030, including 6 goals which are as follows: improving water quality by reducing contamination, eradicating, discarding, and minimizing the release of hazardous substances and materials, halving the proportion of crude effluents, and significantly increasing recycling and safe reuse globally [14]. To achieve this aim, there must be a global focus on reducing urban river pollution through monitoring the quality of discharge from industries and waste stabilization ponds. However, no present rule requires these developing contaminants to be determined in treated wastewater, surface water, drinking water, or the atmosphere. Although drug abuse is now recognized as a global problem [15–17], the secondary effects of these substances have not yet been evaluated, such as their contribution to pharmaceutical load in the environment. The evidence of illicit drugs in waste and river waters is mostly available in developed countries [3, 18–22]. However, there is a scarcity of information, status, and knowledge regarding Oceania, Asia, and Africa, particularly in sub-Saharan Africa and a huge part of the world. The incidence patterns, destiny, and impact on many environmental compartments remain unknown. As a result, additional research is needed to determine their occurrence in waste and surface waters in developing nations to create a safer ecology.

The article "Contribution of Illicit Drug Use to Pharmaceutical Load in the Environment: A Focus on Sub-Saharan Africa" was published in 2022. Journal: J Environ Public Health.

## 2. Illicit Drug Use

Substance abuse, often known as drug abuse, includes using illicit drugs in quantities or with methods that endanger the user or others; it is a type of substance abuse disorder. Society is mostly concerned with the primary effects of drug abuse; this is possibly because the evidence of the effects of addiction and its contribution to the global burden of diseases is available [23–25]. The contribution of drug abuse to the pharmaceutical load and pollution, in general, should not be ignored as these substances may pose an unknown risk to the ecosystem, which may impair its sustainability.

## 3. Current Status of Abuse

Initially, traditional drugs of abuse such as heroin prevailed in the illicit drug scene. Later, other products such as novel psychoactive substances (NPS) and other drugs without restrictions were introduced. NPS have not managed to replace the traditional drugs of abuse completely; therefore, they coexist, complicating addiction treatments [26, 27]. The contribution of COVID-19 pandemic and economic downturn to the negative effects of illicit drugs on the impoverished, marginalized, and vulnerable communities is yet to be determined [1, 2]. However, border restrictions are said to increase the price and decrease purity, which may magnify drug problems. These substances are used singly or as cocktails for different reasons, such as to increase effects, for example, the mixture of prescription of opioids, cannabinoids, and cathinones [28–30]. Reports of the coexistence of these substances in the black market are available [31–35], and information on the possibility of being utilized by similar methods such as inhalation, smoking, and injecting is available [36–40]. Often, the consumers of substances lack awareness of the types of substances they are using and the interrelated risks; this is often because of mislabelling and adulteration of these substances [9, 39, 41–43]. Previous studies reported [31, 44–48] that drug misuse among teenagers and older persons in sub-Saharan Africa and the potential harm it causes are expected to rise until 2050 [49]; this indicates the need for intervention.

## 4. Drug Abuse in Sub-Saharan Africa

Drug abuse problem is increasing in sub-Saharan Africa, with reports of youth engagement in risk behaviour, including injecting and multiple drug use [49–56]. Olawole and colleagues (2018) conducted a systematic review which included 143201 adolescents from sub-Saharan Africa, having an average age of 16 years [55]. Apart from the fact that the incidence of use of any drug among teenagers was 41.6%, a higher rate of 55.5% was observed in Central Africa. It was further observed that depressant abuse was 11.3%, followed by amphetamines at 9.4%, and heroin was the least at about 4% [55]. These results indicate that youth in sub-Saharan Africa abuse multiple drugs, including prescription drugs (PDs), traditional drugs of abuse (TDA) such as cocaine, novel psychoactive substances (NPS), and natural products, and their mixtures as reported by other researchers [47, 57, 58]. The drawbacks of abuse are seen among youth as the mean age of abusers is about 16 years. These are expected to be participating in school activities. Youths are deteriorating, and as a result, the workforce is lost. Instead of youths participating in income-generating activities, they seek addiction treatment for recovery. Therefore, there is a need for a multidisciplinary approach to tackling drug abuse issues.

The article "Contribution of Illicit Drug Use to Pharmaceutical Load in the Environment: A Focus on Sub-Saharan Africa" was published in 2022. Journal: J Environ Public Health.

## 5. Effects of Illicit Drug Abuse

Reports of drug problems are accompanied by vindictive social impacts such as financial difficulties and communal life, the adverse effect on the industry, education, and family life, and its contribution to crime, violence, and homelessness [59–61]. The mode of drug use also contributes to risk factors, for example, injecting drug use becomes a route through which blood-borne virus circulates to the general population. The most-reported effect of illicit substance abuse is addiction, but the possibility of effects on human beings and the ecosystem through the food chain still needs to be investigated.  Figure 1 shows the roots through which human health and the entire ecosystem may be exposed to these substances.

The results of a study by Aghababaei and colleagues revealed the presence of poisonous metals and bacterial contamination in abused drugs. The study pointed out the presence of the greatest quantities of lead (Pb) ranging 63–213 g/g and chromium (Cr) ranging 427–468 g/g in opium samples [62]. Furthermore, the maximum incidence of microbial pollution was observed in opium samples, whereas heroin samples had the lowest [62]. *Clostridium tetani* was the most common microbe in the tested samples, accounting for almost half of all contaminants [62]. These results indicate the possibility of contamination risks to drug abusers, resulting from these substances being produced illicitly and, therefore, a low possibility of following good manufacturing practices.

On the other hand, the reports of combined exposure of a compound itself or its metabolites and mixtures of multiple drugs are missing globally. The effects of pharmaceuticals in the environments have been reported, such as the development of drug-resistant strain, the possibility of giving rise to more toxic metabolites, extinction of species, mammals, aquatic ecosystem, plants, soil arthropods, and toxic effects [63–65]. The reports of poisonous effects of substance use on the environment are required. The effects of a 96-hour exposure to 500 ng/L of cocaine and 20 ng/L of benzoylecgonine or their mixture on *Mytilus galloprovincialis* were examined [12]. The results show that the oxidative status in the gills and digestive glands of the Mediterranean mussels was not altered by exposure to a single component. The dissimilarity is the exposure to a mixture of illicit drugs which modulated the antioxidant activity in the gills but not in the digestive gland of treated mussels [12]. More research studies about the toxicity of illicit drug mixtures are needed to emphasize the risk that these compounds provide to the ecosystems [61]. Apart from direct health risks to users, other illicit drugs contribute to the pollution of our environment, since some are pseudopersistent while others are persistent. Therefore, illicit drugs persist in the environment, while they bioaccumulate, bioconcentrate, and biomagnify through the food chain. These substances have been identified in environmental samples such as soil, tap/groundwater, wastewater, urban rivers, and streams in developed countries [9, 66–75] and some African countries such as South Africa and Tunisia in some matrices. However, information about their presence in environmental compartments of sub-Saharan countries, possible harm to the ecosystem, and contribution to the pharmaceutical load is not certain. The environmental threat created by emerging contaminants and the contribution of drug abuse should not be ignored as they are associated with more risk factors leading to pollution.

The article "Contribution of Illicit Drug Use to Pharmaceutical Load in the Environment: A Focus on Sub-Saharan Africa" was published in 2022. Journal: J Environ Public Health.

## 6. Evaluation of Environmental Illicit Drug Load

The quantity of illicit drugs used by the inhabitants served by the wastewater treatment scheme is estimated using wastewater-based epidemiology (WBE) [76]. In this case, raw wastewater is collected and investigated for the presence of quantifiable biomarkers of drugs, and the amount of licit or illicit drugs consumed by the inhabitants served by the wastewater treatment scheme is back-calculated [76] after taking composite samples of raw wastewater and analyzing them for certain components such as illicit drugs [76]. The total consumption of a drug is calculated using this number plus a correction factor that considers the average excretion rate of a certain drug residue and the molecular mass ratio of the parent drug to its metabolite [76]. The comparison among cities is done by taking the daily values and dividing them by the number of individuals served by the treatment scheme. This value can be articulated in daily amounts (or daily doses) per thousand inhabitants [76]. The improvement of integrity and scalability of this technique is increased by adopting a standardised procedure [77]. It is important to ensure that data from different sources are more reliable and comparable. The Sewage analysis CORe group Europe (SCORE) network conducted its first Europe-wide study in 2011, and its results provided a comprehensive insight into the uncertainties associated with all of these procedures [77]. As a result, the team developed best-practice protocols for sampling, sample handling, chemical analysis, back-calculation, and data reporting. This procedure was refined and updated during successive European analytical campaigns undertaken annually [77]. This technique can complement the current methods as it can be done without inversion of anyone's privacy and can help in region-wise follow-up of drug use.  Table 1 provides the list of reported normalized daily load of selected drugs including illicit drugs.

## 7. Contribution of Drug Abuse to Pharmaceutical Load in the Environment

Illicit drug environmental occurrences are mainly due to human excreta after illicit drug consumption. These substances, like other pharmaceuticals, have biological activity and range from pseudopersistent to highly persistent compounds; hence, they persist in the environment while causing harm to the ecosystem, as other contaminants increase the pharmaceutical load on the environment. However, its contribution is not clear [79–82]. Although the amount of these compounds in the environment is minimal, the dangers to humans and the environment must be addressed. There are reports of growing illicit drug consumption in Sub-Saharan Africa [18–21, 83–87]. The contribution of drug abuse in increasing pharmaceutical load to environmental compartments needs to be thoroughly investigated and ascertained for a greener ecosystem. The contribution of drug abuse to environmental pollution is not clear, but most of these drugs are manufactured illegally in the clandestine laboratory, and the possibility of following good manufacturing practice (GMP) guidelines is low. Therefore, the possibility of waste from clandestine laboratories being discharged into nearby streams or rivers, dumped in the wastewater plant, or utilized in landfills is higher. Through these practices, the possibility of contaminating groundwater is high, increasing the need to monitor illicit drug use by analyzing their presence in the environmental matrices such as soil, wastewater, and surface and groundwater for sustainability. These substances producing toxic by-products are rare, requiring research [88]. Archer and colleagues conducted a two-year study on monitoring emerging contaminants and illicit drugs in the wastewater treatment schemes in South Africa and observed a decrease in active chemical loads during the monitoring period [78].  Table 2 provides the list of comparative active chemicals' (ACs) loads reported from various drug categories.

The article "Contribution of Illicit Drug Use to Pharmaceutical Load in the Environment: A Focus on Sub-Saharan Africa" was published in 2022. Journal: J Environ Public Health.

The reported chemical load from illicit drugs is comparable to anti-inflammatory and antibiotics (Table 2). However, more data are required to initiate guideline reforms to include illicit drugs in environmental assessment and monitoring activities for environmental sustainability.

Illicit drugs have been shown to contaminate aquatic ecosystems worldwide, which has been expected for many years [89–92]. Horky and colleagues revealed fish addiction results in changes in habitat preferences, with unanticipated negative repercussions on individual and inhabitant levels [93]. This may be contributed by the dumping of illegal drugs into freshwater ecosystems or contaminated effluents. Methamphetamine is regarded as one of the most serious worldwide health threats, producing addiction and behavioural changes in brown trout *Salmo trutta* at a concentration of 1 *µ*gL^−1^ [93]. The impact of these substances may be amplified through bioaccumulation, bioconcentration, and biomagnification through the food chain, indicating the possibility of harming ecosystems. When consumed in a food chain, these contaminated fish may cause health problems, including addiction to nonabusers. These compounds may also lead to transformational and disinfection products as other contaminants that may further impact ecosystem sustainability.  Figure 2 shows the structure of methadone and its disinfection by-product.

The environmental impact of remnants of active chemicals from contraceptive pills includes the feminization of male fish downstream, resulting in a deteriorating fish population [94–96]. Few reports on misuse of oral contraceptive pills (OCPs) for topical use such as to increase hair growth and give negative findings for addictive drug screening tests are available [97]. Increased topical use of OCPs may throw the ecosystem off balance and lead to an unsustainable environment. Pharmaceutical drug methadone, which is used to mitigate addiction caused by the recreational use of opioid heroin, was observed to create N-nitrosodimethylamine (NDMA) in surface and wastewater due to the application of chlorination as a disinfection technique [88]. A probable human carcinogen reaches drinking water after formation as disinfection by-products, and its threshold in drinking water is 7 ng/L according to USA guidelines [88]. The evaluation and monitoring of these contaminants are important for the safety of the ecosystem.

The article "Contribution of Illicit Drug Use to Pharmaceutical Load in the Environment: A Focus on Sub-Saharan Africa" was published in 2022. Journal: J Environ Public Health.

## 8. Challenges of Sewerage Systems in Sub-Saharan Africa

It is observed that over 50% of the world's population lives in urban areas [20], individuals living in slums are increasing by about 20 million each year, and people living in metropolitan areas lack proper sanitation. The sewage system in sub-Saharan Africa faces difficulties, since it was not intended to handle emerging contaminants [66] such as pharmaceuticals and drug abuse. Therefore, these substances remain in the wastewater after treatment and are released into the environment. Another challenge is faecal sludge management (FSM). In most settings, the sludge is utilized as an organic fertilizer, as the facility is incapable of removing or not designing the sludge also is contaminated. Urban cities in sub-Saharan Africa lack the proper FSM approach, and most cities do not prioritize FSM. FSM is considered an insignificant aspect of environmental sanitation, and discharging FS in water bodies, lagoons, and the environment is regularly considered the normal and proper way of dealing with FS. At the same time, through the utilization of sludge in the reclamation of agricultural land or fertilizer contaminants, their metabolites and transformation products [98] are circulating in the environment [73, 99–102]. These substances are toxic; hence, the possibility of causing harm to humans or the environment is rising. Another issue confronting wastewater treatment plants in sub-Saharan Africa is the lack of modern, state-of-the-art facilities for contamination identification and quantification. This issue will significantly be observed in drug of abuse as traffickers and manufacturers change precursors and drug design to avoid legal constraints concerning their manufacture, sale, and use [47, 48].

## 9. Global Occurrences of Illicit Drugs in Environmental Compartments

Tendencies of encountering drug abuse and other drugs in the environment are increasing, and this threat is recognized as an issue of concern. Researchers employed wastewater analysis to track the pollution produced by these compounds in the environment and assess the efficacy of treatment plants in removing them [19, 103, 104]. Sources, behaviour, and fate of chemicals in the environment as singly have been investigated broadly [105, 106]. The current research indicates the existence of these drugs in mixtures such as drug abuse and other prescription drugs, which may result in toxicity due to drug-drug interactions or combined concentration for a drug with a similar mode of action. Reports of global occurrences of illicit drugs in wastewater effluents, influents, and urban rivers are available [18, 19, 40, 42, 53, 107–115].  Table 3 provides data on the prevalence of illicit drugs around the world. As millions of people abuse amphetamine-like stimulants, marijuana, cocaine, heroin, and other substances, the volumes of illicit drugs used worldwide may be equivalent to those of prescriptive drugs. Therefore, to control and monitor our environment, drug abuse should be kept under consideration as these substances are among emerging contaminants [17, 104, 116].

The article "Contribution of Illicit Drug Use to Pharmaceutical Load in the Environment: A Focus on Sub-Saharan Africa" was published in 2022. Journal: J Environ Public Health.

In most of the areas provided in Table 3, the load increased on Saturday and Sunday. This might be because the number of residents increased in participating in recreational activities. As a result, more people consume drugs, possibly more doses because there is no work, and others may come from far areas for recreation.

## 10. Occurrences of Illicit Drugs in African Environmental Compartments

Reports of drug abuse in South Africa are available [117–122], and the increased crime rate has been associated with drug abuse apart from other factors [118, 119]. Identification of multiple drugs, including TDA and NPS, indicates polydrug nature and the possibility of contamination of the ecosystem. This study also shows that the possibility of the availability of clandestine laboratories in the area or reported MDMA and HMMA is from clandestine sources. This is because both are chiral with conventional manufacturing methods [123]. The list of identified illicit drugs in South African wastewater is provided in Table 4.

## 11. Tunisia

Identification of illicit drugs in wastewater confirms their use, informs their presence in the environment, and the possibility of harm to the ecosystem. Multiple drugs indicate the polydrug nature of abuse and the existence of TDA and NPS in the black market requires intervention. The most significant aspect is that these compounds are introduced into the environment, increasing the pharmaceutical load and decreasing ecosystem safety.  Table 5 provides the list of identified illicit drugs in northern Tunisia.

## 12. Occurrences of Illicit Drugs in Sub-Saharan Africa Environmental Compartments

In Sub-Saharan Africa, the evidence on the existence of illicit drugs, their metabolites, and transformation products is not sufficient. For example, it has been revealed that there are few reports on the presence of illegal drugs, metabolites, and transformation by-products in the environment of several sub-Saharan African countries. Officials are concerned with potential harm to human beings and the environment due to their toxicity, by itself or in combination [60, 126, 127]. The scarcity of information is contributed by the fact that some of these countries lack state-of-the-art laboratory facilities for their identification and quantification [128]. Therefore, there is a need for monitoring authorities and policymakers to ensure the availability of these types of equipment for analysis of emerging contaminants, including drug abuse, for a safer ecosystem.

The article "Contribution of Illicit Drug Use to Pharmaceutical Load in the Environment: A Focus on Sub-Saharan Africa" was published in 2022. Journal: J Environ Public Health.

## 13. Circulation of Drugs of Abuse in the Ecosystem

In the 1970s, countries in Europe and the United States developed nearly full sewer networks and wastewater treatment plants (WWTPs), putting a stop to the practice of directly discharging sewage into metropolitan waterways [129]. This halted the decline of many urban rivers' water quality, gradually improving [129, 130]. At the start of rapid urbanization in the 1980s, China experienced major pollution due to a big amount of sewage being immediately released into rivers; the same was true in most other developing countries [129]. So far, most African governments, mostly in sub-Saharan Africa, have not restricted sewage discharge straight into urban rivers and other environmental compartments [100–102]. In the sewage based on the design of sewage treatment, there is the possibility of further transformation of these substances, possibly into more toxic by-products. The majority of these illicit drug residues have powerful pharmacological activity, and their existence in aquatic settings might have serious consequences for human beings and the ecosystem.  Figure 3 shows the structure of the illicit drug heroin and its metabolites which may further be converted into transformational by-products due to treatment conditions or environmental conditions.

Mostly identified drugs such as ecstasy, methamphetamine, MDA, morphine, and cocaine have powerful activity, and their presence in surface waters as complex mixes with residues of innumerable drugs may result in unforeseen pharmacological interactions, with hazardous consequences on the aquatic ecosystem, as reported by other researchers [13, 18, 42, 60, 61, 73, 86, 131, 132]. In the ecosystem, these substances may bioaccumulate, bioconcentrate, and biomagnify through the food chain, as shown in Figure 1. When humans consume food, these substances may enter into a human being and create possible harm, especially to nonabusers.

## 14. Conclusions

Apart from the basic repercussions of drug abuse, which include chronic diseases such as cirrhosis, heart disease, blood-borne bacterial and viral infections, and mental problems indicating contribution to the global burden of diseases [23–25], the contribution of drug addiction to the degradation of the environment and biodiversity loss must be considered. Illicit drugs such as opioids were observed to be contaminated with heavy metals and microorganisms [62]. Reports of environmental and ecosystem contamination by illicit drug use are available, including addiction in fish as a result of methamphetamine exposure [93], which indicates the possibility of development of addiction to nonabusers through the food chain. Therefore, the development of an unsustainable ecosystem needs intervention. These results indicate the possibility of drug abuse contributing to contamination and exposure to contaminants and possible harm. In this case, studies on environmental effects of drug abuse need to be conducted singly and in combination to evaluate the contribution of illicit drug use to environmental contamination for conservation and sustainability of the ecosystem.

The article "Contribution of Illicit Drug Use to Pharmaceutical Load in the Environment: A Focus on Sub-Saharan Africa" was published in 2022. Journal: J Environ Public Health.

## Figures and Tables

**Figure 1:** Description of possible illicit drug exposure to the ecosystem through the food chain. This figure indicates that human beings act as sources and sinks of these contaminants. The possibility of the clandestine laboratory releasing contaminated effluents into the environmental compartments is higher than that in treatment schemes which may magnify the problem.

**Figure 2:** Structural representation of 6-(dimethylamino)-4,4-diphenylheptan-3-one and NDMA, its disinfection by-product.

**Figure 3:** Structure of heroin and its metabolites which may further be changed to transformational by-products due to environmental and treatment conditions.

**Table 1:** Reported normalized daily load of selected drugs, including illicit drugs.

Active chemical	NDL, mg/day/1000 inhabitants	References
Codeine	71.1–441	
Caffeine	831.7–3094.9	
Acetaminophen	785–9953.5	[78]
Diclofenac	21.7–94.1	
Naproxen	35.1–141.3	
Sulfamethoxazole	384.4–741.6	
Carbamazepine	30.1–143.1	

**Table 2:** Comparative active chemicals (ACs) loads reported from various categories of drug.

Drug category	Daily load in g/day	References
Anti-inflammatory	100–3000	[78]
Anticonvulsant	0–100	
Anticorrosive	100–200	
Opioids	0–500	
Illicit drugs	800–3800	
Antibiotics	500–4200	

**Table 3:** Representatives of instances of illegal substances and their metabolites in environmental compartments around the world.

Country	Illicit drug	Consumption (mg/day/1000 inhabitants)	References
Hong Kong	Ketamine	1400–1600	[117]
	Cocaine	160–180	
	Methamphetamine	180–200	

Europe	Cocaine	0–2000	[21]
	Amphetamine	LOQ–3040	
	Methamphetamine	50–400	
	MDMA	LOD–615	
	THC-COOH	25–200	

Brussels (Belgium)	Cocaine	400–650	[43]
	Heroin	350–400	
	MDMA	5–25	
	Methamphetamine	0–5	
	Amphetamine	40–80	

South Korea	Methamphetamine	14.9–28.6	[3]
	cis-Tramadol (opioid)	27.5	

UK	MDMA	50	[116]
	Methamphetamine	110	
	Benzoylecgonine	1000	
	Mephedrone	50	
	06-MAM	80	
	Ketamine	200	
	Amphetamine	120	
	Cocaine	1500	

06-MAM, 6-monoacetylmorphine; MDMA, 3,4-methylenedioxymethamphetamine; THC; tetrahydrocannabinol.

The article "Contribution of Illicit Drug Use to Pharmaceutical Load in the Environment: A Focus on Sub-Saharan Africa" was published in 2022. Journal: J Environ Public Health.

**Table 4:** Identified illicit drugs in South African wastewater.

Substance	Illicit drug (mg/day/1000 inhabitants)		References
	WWT1	WWT2	
MDMA	0–2.23	0.5–65	
Methamphetamine	15–45	140–250	
Mephedrone	-	7.6	
06-MAM	-	2.09–5.54	
Cocaethylene	0–16	5–80	[124]
Cocaine	2–6	10–40	
Benzoylecgonine	6–17	38–78	
Amphetamine	0.7–1.4	4–12	
HMMA	0–0.25	0.7–2.5	

MDMA, 3,4-methylenedioxymethamphetamine; 06-MAM, 6-monoacetylmorphine; Bdl, below detection limit; WWT, wastewater treatment.

**Table 5:** Identified illicit drugs in northern Tunisia.

Substance	Illicit drugs (mg/day/1000 inhabitants)	References
Amphetamine	LOQ–79	
MDMA	LOD–51	
Methamphetamine	LOD–24	
Benzoylecgonine	LOQ–450	[125]
Mephedrone	LOQ–102	

## Data Availability

The data used to support this study are included within the article.

## Abbreviations

AMR: Antimicrobial resistant
ACs: Active chemicals
BFRs: Brominated flame retardants
BE: Benzylecgnonine
COC: Cocaine
ECs: Emerging contaminants
COVID-19: Coronavirus disease-19
DOA: Drug of abuse
FS: Faecal sludge
FSM: Faecal sludge management
LOQ: Limit of quantification
LOD: Limit of detection
MDMA: 3,4-Methylenedioxymethamphetamine
06-MAM: 6-Monoacetylmorphine
NPS: Novel psychoactive substances
NDMA: N-Nitrosodimethylamine
PFCs: Perfluorochemicals
PDs: Prescription drugs
TDA: Traditional drug of abuse
UNODC: United Nation Office on Drug Control
WWTPs: Wastewater treatment plants.
